The article "White Matter Injury: An Emerging Potential Target for Treatment after Subarachnoid Hemorrhage" was published in 2023. Journal: Oxid Med Cell Longev.

# White Matter Injury: An Emerging Potential Target for Treatment after Subarachnoid Hemorrhage

**DOI:** 10.1155/2023/3842493

**Published:** 2023-02-07

**Authors:** Yibo Liu, Yezhao He, Jiahao Zhang, Xiaoyu Wang, Anke Zhang, Qian Yu, Kaikai Wang, Yuanjian Fang, Qingsong Jiang, Sheng Chen

**Affiliations:** ^1^Department of Neurosurgery, The Second Affiliated Hospital, School of Medicine, Zhejiang University, Hangzhou, Zhejiang Province, China; ^2^Key Laboratory of Precise Treatment and Clinical Translational Research of Neurological Diseases, Hangzhou, Zhejiang, China; ^3^Department of Neurosurgery, Quzhou Kecheng People's Hospital, Quzhou, Zhejiang Province, China

## Abstract

Subarachnoid hemorrhage (SAH) refers to vascular brain injury mainly from a ruptured aneurysm, which has a high lifetime risk and imposes a substantial burden on patients, families, and society. Previous studies on SAH mainly focused on neurons in gray matter (GM). However, according to literature reports in recent years, in-depth research on the mechanism of white matter (WM) is of great significance to injury and recovery after SAH. In terms of functional recovery after SAH, all kinds of cells in the central nervous system (CNS) should be protected. In other words, it is necessary to protect not only GM but also WM, not only neurons but also glial cells and axons, and not only for the lesion itself but also for the prevention and treatment of remote damage. Clarifying the mechanism of white matter injury (WMI) and repair after SAH is of great importance. Therefore, this present review systematically summarizes the current research on WMI after SAH, which might provide therapeutic targets for treatment after SAH.

## 1. Introduction

Subarachnoid hemorrhage (SAH) is identified as a subtype of stroke with high morbidity and mortality which is mainly caused by a ruptured aneurysm [1]. Considerable advances in the management of aneurysmal SAH have reduced the risk of morbidity and mortality in recent years [2]. Although acute management can obtain an immediate effect to save lives and reduce disability rates, it cannot stop or reverse brain injury. In both clinical and basic studies, it was widely reported that neurological deficits and cognitive impairments were exceedingly common after SAH [3].

Reviewing previous studies of SAH, we could find that most of the studies on brain injury after SAH were concentrated on gray matter (GM). Although white matter (WM) accounts for approximately 40% of the human brain volume, white matter injury (WMI) associated with SAH is a relatively poorly investigated field that has only recently begun to be addressed in more detail [4–6]. After SAH, WM is massively damaged, which not only causes various dysfunctions or disabilities but also causes dysfunction in the remote nerve projection area. By inhibiting or reducing WMI, it can limit the scope and extent of SAH and reduce clinical symptoms [7]. Measures to promote WM regeneration and remodeling are beneficial to functional recovery during the rehabilitation period. Clarifying the mechanism of WMI and repair after SAH is of great significance and can provide new strategies for SAH treatment. Therefore, we summarize recent basic and clinical SAH research concerning WMI.

## 2. Characteristics of White Matter

The human brain is comprised of both GM and WM. According to neuroimaging studies, the volume of WM is 456 ± 48 cm^3^ in men and 392 ± 42 cm^3^ in women, which accounts for 40% of the total human brain volume [8]. WM mainly contains long extensions of myelinated and unmyelinated axons that are organized into tracts and surrounding glial cells and blood vessels. WM is classified into periventricular WM and deep WM based on anatomical location. Periventricular WM is found immediately adjacent to the ventricles whereas deep WM is distinctly isolated from the ventricles and found beneath the cortex [9].

Similar to GM, WM is vulnerable because of many characteristics: (1) WM has lower blood flow than GM. And there is little collateral circulation, especially in deep WM. (2) The autoregulation of blood vessels in the WM area is worse than that in the GM area. (3) Certain areas of normal WM, especially the blood-brain barrier around the ventricle, have inherent fragility. Blood-derived macrophages can also invade adjacent ventricles. (4) The WM area is rich in acute and chronic inflammatory glial cells, and the subsequent inflammatory response is intense. (5) Oligodendrocytes, especially oligodendrocyte progenitor cells (OPCs), are highly sensitive to ischemia-induced oxidative stress, excitotoxicity, and inflammation, which contribute to OPC death and WMI after brain injury. When brain tissue is damaged, even if only a single oligodendrocyte is damaged, it may cause damage to multiple neuron axons, thereby affecting neurological function [10] (Figure 1).

## 3. The Relationship between WMI and SAH

### 3.1. SAH: A Cause of WMI

There are two distinct physiological insults that occur immediately after SAH: (1) sudden bleeding into the subarachnoid space and (2) hypoxia due to disturbed cerebral circulation and increased intracranial pressure [11]. Both of these two initial changes and subsequent pathophysiological mechanisms are the fatal blow to the vulnerable white matter. Among the subsequent pathophysiological processes, neuronal injury is the major pathophysiological event in SAH. Axons in the WM consist in the integrity of neuronal function. Both evidence in SAH patients and animal models have revealed that abnormal WM signals can be observed with MRI in the early stage after SAH [12], even in the hyperacute phase (within 4 h) [13], indicating the existence of WMI. Moreover, autopsied cases of SAH found apparent WM lesions separate from prevalent cortical and hypothalamic lesions [14] and also showed remarkable edema and congestion in the deep part of frontal WM and severe diffuse axonal injury [15].

### 3.2. WMI: A Predictor of SAH

Mild WMI results in long-term functional, neurocognitive, and emotional symptoms. Damage to different WM tracts is associated with a patient's specific symptoms, such as attention deficits, memory problems, and deficits in executive functions. The overall burden of WMI is related to both speed of information processing and overall functional outcome [16, 17].

Both experimental and clinical research demonstrated that WM lesions in the acute phase are associated with poor outcomes [18, 19]. In the clinic, SAH patients who initially present with low World Federation of Neurosurgical Societies (WFNS) grades and hydrocephalus (which may be the reason for WM damage) can be efficiently treated with extraventricular drainage and often show rapid improvement, but patients with high-WFNS grades and low-Glasgow Coma Scale scores rarely have good recoveries [20].

## 4. Identification and Monitoring of WMI

### 4.1. Histological Changes

In 1989, the autopsy reports of six SAH cases indicated considerable congestion and edema in the deep frontal WM, as well as axonal degeneration under microscope examination [15]. After SAH, axonal injury appeared in the subcortical WM region. Electron microscopy showed abnormalities in the myelin sheath, axon membrane, mitochondria, and axon cytoskeleton, including disorders and dissolution of the myelin sheath structure. The number of microtubules was reduced or completely lost, nerve filament spacing shrank, dense clustering occurred, axonal membrane segment was separated from the inner layer of the myelin sheath to expand the axon and myelin space, and mitochondrial swelling occurred, and these changes in the axon were consistent with the literature [21–23].

For experimental research, studies show long-term WM loss after SAH in mouse and rat models and found histological changes 7 days after SAH. A comparison of corpus callosum thickness of both hemispheres indicated WM thinning ipsilateral to the SAH induction site [4, 24]. However, WMI measured as MBP loss was only observed in severely affected SAH animals and was not detectable in mildly affected SAH animals. Moreover, loss of MBP staining was clearly less severe than gray matter damage, measured as MAP 2 loss. These data indicate that WM damage could result as a consequence of neuronal damage [4].

### 4.2. Imaging Changes

MRI has reliability and well-documented advantages compared with CT in detecting cerebral edema, white matter injury [5, 25, 26], ischemic lesions [27, 28], and acute hydrocephalus [29–31]. Imaging in the acute phase of SAH may lead to better delineation of the EBI caused by SAH. However, MRI is usually not used in the acute phase of SAH as patients require critical care monitoring, and MRI requires longer imaging time with minimal clinical monitoring [32, 33].

MRI is a noninvasive technique that can provide a three-dimensional assessment of metabolism, tissue morphology, and function and has been widely applied to display the architecture and function of WM [34]. Due to the differences in water content and myelination, T1, T2, and fluid-attenuated inversion recovery (FLAIR) sequences used in conventional MRI can accurately distinguish GM and WM [35] and measure the volume of WM [36]. In theory, the volume of WM represents the quantity of axons, their diameter, the thickness of the medullary sheath, and their compactness [37]. WMI presents as WM hyperintensities on T2-weighted or FLAIR sequences and hypointensities on T1-weighted images relative to normal white and gray matter.

A retrospective quantitative MRI study indicated diffuse vasogenic edema and WMI after SAH [38]. For long-term outcomes, the researchers found progressive axonal damage after 12 months, compared with three weeks of magnetic resonance imaging in patients with good-grade SAH that colocalized with iron accumulation [39]. Knowing the temporal change in CC T2 hyperintensity is quite important in determining the time frame of maximal injury and optimizing the window for therapeutic intervention and thereby prompting a better outcome [40].

In animals subjected to SAH by endovascular perforation, signs of WMI were observed as evidenced by marked hyperintensity of the corpus callosum and/or external capsule assessed by T2WI [5]. SAH rats in the severe state had large T2 lesions, worse neurological outcomes, and higher incidence of hydrocephalus and WMI compared to the mild stage [18]. 57% of WT mice with SAH had unilateral WM T2 hyperintensity area, the opposite side to the endovascular perforation, at 4 hours after SAH [13]. In addition, the data of T2 hyperintensity in WM is found bilaterally at 24 hours after SAH and improved by the late acute phase (8 days) [5, 40, 41]. Hyperacute T2 hyperintensity lesion of the opposite side of perforation might be a contrecoup injury caused by physical compression from the subarachnoid blood. Then, a hypoxic state causes bilateral WMI in the brain. Alternately, there may be differential access of subarachnoid blood to the left and right lateral ventricles causing differential injury [13].

DTI can detect the magnitude and directionality of water molecules in live tissue and is more sensitive than conventional MRI in detecting WMI [34]. In contrast to GM, water in WM moves swiftly along the direction of the axon due to the axonal tract, while myelination inhibits water movement vertical to the fasciculation, presenting a high fractional anisotropy (FA) value [42]. By using DTI, many studies have reported SAH-related neural tract injuries [43–55]. Researchers have reported injury of the lower portion of the ascending reticular activating system between the pontine reticular formation and the thalamus in patients with SAH by using DTI [50]. Another study has done fiber tracking and DTI for 11 patients with ACoA aneurysm rupture who had sustained memory impairment and found decreased FA values and absent trajectory of the cingulum and the fornix [44]. Moreover, small-sample clinical experimental results suggested that DTI parameters, including FA and apparent diffusion coefficient, in WM areas are associated with SAH prognosis [56, 57].

In conclusion, MRI is not routinely used for initial assessment and follow-up imaging in patients after SAH, likely because of longer imaging time, uncertainty regarding feasibility, and potential adverse events of MRI in SAH patients. Increasing studies support the use of MRI as a safe and clinically valuable with well-documented advantages in detecting WMI, ischemic lesions, cerebral edema, acute hydrocephalus, and so on. The available information is quite important in leading to better delineation of the early brain injury caused by SAH and optimizing the window for therapeutic intervention and thereby prompting a better outcome. Establishing imaging criteria for the diagnosis of WMI after SAH may help quantitatively evaluate the severity of WMI and the effectiveness of treatment interventions.

### 4.3. Biomarker Changes

Neurofilament light chain (NF-L) is a major component of the axonal cytoskeleton [58]. Research demonstrates that NF-L can be detected in CSF within 24 h after SAH. The release of NF-L into the CSF has not been determined definitively, but possibilities include axonal shear injury due to a rapid pressure wave occurring at the time of aneurysm rupture, an acute rise in intracranial pressure causing mechanical deformation of axons, transient global ischemia, or ischemic WMI due to microvascular dysfunction [59].

The hypothesis of ongoing axonal damage in patients with aSAH is furthermore supported by the report of sustained elevation of CSF total-tau. The study showed that high total-tau levels were associated with poor functional outcomes (modified Rankin scale ≥ 4) at 1 year after aSAH. A similar association was found with 3/5 neuropsychological tests indicative of impairments in cognition, psychomotor speed, visual conceptualisation, and frontal executive functions 12 months after aSAH. These results suggest that protein tau merits further study in the context of aSAH possibly serving as a biomarker for axonal injury as well as possibly predicting morbidity and mortality following aSAH [60].

Increased calpain- and caspase-3-mediated spectrin breakdown products (SBDPs) are found in a number of acute and subacute neurodegenerative conditions [61–63]. Research suggested SBDPs as useful biomarkers of axonal injury and WMI [64]. The clinical study found that both calpain- and caspase-mediated SBDP levels are significantly increased in patients suffering from aneurysmal subarachnoid hemorrhage. The concentration of SBDPs in CSF was found to increase significantly over the baseline level up to 12 hours before the onset of cerebral arterial vasospasm [65]. Persistent elevation of SBDPs might be associated with cerebral infarction and/or overwhelming axonal injury resulting in death.

Myelin basic protein (MBP), a primary component of the myelin sheath, is a marker of demyelination of the white matter [66]. The experimental study showed long-term white matter loss visualized by immunohistochemistry for MBP at 21 days post-SAH in a rat model [4]. For clinical research, researchers have observed significantly higher levels of MBP on days 0–3 post-SAH in patients following surgical intervention and with large ICH compared with no intervention and small ICH/no ICH. The early MBP levels also correlated with the treatment outcome and with the ICH volume [67]. Moreover, CSF MBP is an indicator of the severity of brain damage in SAH patients. CSF MBP concentrations remained at higher levels than the upper limit of normal during the period when measurements were performed [68].

To sum up, effectively using biomarkers of WMI in CSF or blood after SAH could improve strategies for diagnosing and advancing the ability to monitor the efficacy of treatments. Therefore, further studies are needed to find more easily available and detectable biomarkers of WMI after SAH and confirm the sensitivity and specificity of these biomarkers.

## 5. Mechanisms

Since most blood is released into the subarachnoid space without direct nervous tract disruption, WMI after SAH was considered to be the consequence of pathological mechanisms (Figures 2 and 3).

### 5.1. Elevated Intracranial Pressure

Approximately 50-85% of SAH patients are caused by a ruptured aneurysm. When aneurysm ruptures, blood entering the subarachnoid space can result in a sharp elevation in intracranial pressure (ICP) [1], which may also form a mechanical pressure to deep WM, also leading to SAH-associated WMI, especially in the region distant from the rupture point [19, 25, 69]. Early decompressive craniectomy has been proven to play an important role in improving both the motorial and cognitive prognoses of SAH patients. This may be due to the reduction of WMI caused by the biomechanics of ICP after SAH, but further research is needed to confirm this hypothesis [6, 70].

### 5.2. Ischemia

The brain accounts for only 2–3% of body weight, but the blood supply of the brain is approximately 20% of the heart output, and the brain has virtually no excess oxygen and glucose reserves [71]. WM has lower blood flow than GM, and there is little collateral circulation, especially in deep WM [72]. Furthermore, oligodendrocytes, especially oligodendrocyte progenitor cells (OPCs), are highly sensitive to ischemia-induced oxidative stress [73], which contribute to OPC death and WMI after SAH. Importantly, WM becomes more susceptible to ischemia with age [74]. In summary, WM is highly vulnerable to ischemia and is often injured more severely than GM.

ICP increase, vascular constriction, and microcirculation thrombosis can lead to extensive cerebral ischemia after SAH [6]. MRI scanning detected a significant T2 hyperintensity signal in the WM region revealing that cerebral blood flow was significantly reduced in WM after SAH [75]. And researchers also found that, even in good-grade SAH patients, the incidence of elevated ICP was associated with a lower blood perfusion level in the WM region after SAH [69].

### 5.3. Hydrocephalus

Hydrocephalus has been reported to occur in 6%–67% of patients with subarachnoid hemorrhage (SAH). When SAH occurs, blood coagulation and by-products in subarachnoid granulation can block the outflow tract of CSF causing severe hydrocephalus. Approximately 20%–30% of patients with SAH are known to have a permanent impairment of CSF conversion [76, 77]. This condition can lead to unfavorable neurologic function and deterioration in functional outcomes [1].

The study shows that acute communicating hydrocephalus occurs simultaneously in the mouse endovascular puncture model of SAH. The onset of hydrocephalus was rapid and sustained, occurring within 6 h of SAH and remaining present for at least 72 h [78]. Acute hydrocephalus after SAH reduces cerebral perfusion and mainly affects deeper areas of the brain, specially periventricular white matter (PVWM) in the brain [79, 80].

### 5.4. Blood-Brain Barrier Damage

Blood-brain barrier (BBB) disruption is recognized as a key mechanism of WMI in various central nervous system diseases that often occur early in the disease and contribute to promoting consequent WMI at a later time point [81, 82]. It is also known that BBB disruption is an important pathology of early brain injury and a risk factor for worse outcome after SAH [83].

Transmission electron microscopy showed ultrastructural abnormalities in WM microvessels, including swollen astrocyte endfeet with autophagosomes, tight junction detachment, erythrocyte trapping within vessel lumens, and basement membrane irregularities. These results clearly demonstrate that BBB disruption occurs acutely in WM following SAH [41].

Studies showed that T2 hyperintensity was more prominent in WM than in other cerebral regions 24 hours after SAH, and this was consistent with albumin leakage detected by immunostaining [26, 41]. Moreover, at 4 hours after SAH, even animals without T2 hyperintensities already had albumin leakage. This result suggests that BBB disruption starts very soon after SAH onset before MRI changes and that those areas evolve into T2 hyperintensity lesions [13].

Researchers recently examined BBB leakage and brain endothelial tight junction protein changes in a similar endovascular perforation model of SAH but in rats. They found evidence of BBB disruption with an early opening as early as 30 minutes that peaks at 3 hours and a later disruption that peaks at 72 hours post-SAH. Those results were mirrored by changes in the brain endothelial tight junction proteins, occludin and ZO-1 [84].

In basic research, researchers reported that MMP-9-induced BBB disruption contributes to WMI after SAH. In addition, increased secretion of MMP-9 from astrocytes and oligodendrocyte precursors caused a disruption of the blood-brain barrier (BBB) and subsequent WMI following SAH [41]. Furthermore, researchers found that endogenous ApoE increased as early as 6 h after SAH, and APOE deficiency induced a greater production of IL-1*β* which was previously shown to activate MMP-9 and cause BBB disruption [85].

Another study recently reported a significant increase of LCN2 expression in the WM at 24 h after SAH was confirmed, and LCN2 receptor 24p3R was expressed in oligodendrocytes and BBB components. These results suggest that LCN2 might exert effects on these cells through its receptor and contribute to SAH-induced BBB disruption [26]. Actually, LCN2 has the potential to preserve MMP-9 activity by preventing its degradation [86], and there is a close relationship between LCN2 expression and MMP-9 activity in a mouse model of breast cancer [87]. Similarly, the activity of MMP-9 in the WM after SAH is significantly lower in LCN2 knockout mice than in WT mice [41]. But the effect of LCN2 on MMP-9-related pathogenesis, such as BBB disruption after SAH, needs further investigation.

### 5.5. Inflammation and Microglia Response

Evidence showed that neuroinflammation plays a pivotal role in the pathophysiological process after SAH and contributes to early WMI [88, 89]. A recent study revealed APP accumulation and loss of MBP in the WM after SAH, which may have been due to NLRP3 activation and downstream caspase-1 and IL-1*β* in microglia and the induction of apoptosis in oligodendrocytes. A dose of 150 mg/kg MLT inhibited NLRP3 expression, protected WM fibers, and improved neurological scores, indicating that targeting WM protection may be potentially beneficial to patients who experience SAH [90].

Moreover, neuroaxonal injury coincided with the accumulation of activated microglia, reaching its maximum extent between days 7 and 14 after the bleeding, both in murine and human samples [91]. Thus, proinflammatory and prooxidative microenvironment associated with microglial activations may be critical for WMI progression in the settings of SAH [19]. Microglial depletion by CLP pretreatment significantly suppressed the WMI at 24 h after SAH, characterized by better preservation of normal myelin marker MBP and less axonal injury markers of APP and SMI32. In spite of its significant benefits on WMI reduction in the early phase postexperimental SAH, complete microglial depletion, however, may not represent a reasonable therapeutic strategy to be applied in the clinical setting [92]. Actually, in experimental SAH animals and clinical SAH patients, the activated microglia had been reported to act as a double-edge sword. Upon stimulation and activation, microglia polarized to M1 or M2 phenotypes with distinct functions of proinflammatory and immunosuppressive, respectively [93]. A study demonstrated that a BBB permeable apoE-mimic peptide COG1410 promoted M2 microglial polarization through LRP1 activation, leading to less brain edema and WMI as well as neurological deficits in a rat model of SAH [92].

### 5.6. Oligodendrocyte Response

Oligodendrocytes form myelin sheaths, which are essential for axons because they provide nutritional support and guarantee high-speed electrical impulse transmission [94]. Oligodendrocytes have long been thought to be the most vulnerable cells in the CNS in pathological conditions [95]. Myelin sheaths are also susceptible to multiple neurological disorders and lead to motor dysfunction, cognitive deficits, and other neurological impairments [96]. SAH caused significant oligodendrocyte death in the ultra-acute and acute phases which, for mature oligodendrocytes, persisted into the late acute phase [40]. Interestingly, these temporal changes in oligodendrocytes are consistent with the changes in T2 hyperintensity observed on MRI suggesting that oligodendrocyte death may contribute to CC edema. This is relevant from a clinical perspective as global cerebral edema is an independent risk factor for worse outcomes after SAH [97]. Researchers speculated a possible mechanism in which, after the onset of SAH, a rapid degeneration and demyelination of WM occur accompanied by a decrease in MCT1 in oligodendrocytes in the WM region, which interferes with the energy supply of oligodendrocytes to axons and aggravates WMI [98]. Another study discovered that LCN2 knockout exerts a protective role, reducing oligodendrocyte and oligodendrocyte progenitor cell death on day 1 after SAH. This result suggested that LCN2 may be involved in oligodendrocyte death after SAH [40].

Oligodendrocyte progenitor cells (OPCs) are the main source for repairing damaged oligodendrocytes and a population of cells that maintain WM homeostasis and participate in long-term WM repair after injury [99, 100]. Therefore, as the damage occurs, OPCs are recruited to the lesioned area, where they differentiate into mature remyelinating oligodendrocytes and engage in the formation of new myelin sheaths around axons [101]. Actually, after SAH, OPCs decreased during the ultra-acute and early acute phases; they recovered in number by the late acute phase [97]. Recent study found that OPC proliferation and migration occurred after SAH and determined that these processes were related to remyelination. Nexilin was demonstrated to be a key molecule regulating OPC migration which can serve as a therapeutic target for the acute stage of SAH-induced demyelination [102]. Another experimental study found that inhibition of LCN2 promotes remyelination and myelin maturation after WMI. Moreover, LCN2 inhibits OPC differentiation by mediating the receptor SCL22A17 and downstream transcription factor EGR1 [103].

### 5.7. Iron

Iron is transported into the extracellular fluid of CNS under healthy conditions, through receptor-mediated endocytosis of the brain capillary endothelial cells and subsequently, which is less clear, into the brain extracellular fluid where it is found unbound and transferrin-bound. Iron is then taken up by neurons, oligodendrocytes, and astrocytes [104]. Following SAH, the brain is exposed to high concentrations of hemoglobin and its downstream products not only on the surface of the brain but also in deeper layers of the cortex. Although iron is an essential cofactor for myelination, synthesis of neurotransmitters, and neuronal development, free iron can lead to oxidative stress and neuronal cell damage through radical formation secondary to Fenton reactions [105, 106].

Clinical research provides evidence that the location of iron deposition was associated with microstructural disintegration of the WM tracts adjacent to the midcingulate gyrus at 12 months post-SAH [39]. Moreover, iron levels are elevated in the WM remotely from the bleeding source and constantly increase over time after SAH [107]. These results suggested that iron accumulates in the WM already in the acute phase after SAH, is associated with mechanisms of secondary brain injury, and may be trapped in the brain tissue for a prolonged time after SAH. However, another clinical research observed iron deposits in the cortical gray matter but not white matter at 6 months after SAH which was measured by magnetic susceptibility of brain tissue [108]. Therefore, the process and location of iron deposition after ictus of SAH need further investigation.

The recent experimental studies found that protein levels of hemoglobin scavenger receptor CD163 and HO-1 were highly expressed in WM at the acute stage after SAH [18, 109], indicating that iron overload may be a leading cause of WMI. Another study found that WM LCN2 expression was markedly increased after SAH, and acute WMI was less in LCN2^−/−^ animals [5]. LCN2 is a mediator of iron uptake and could be reduced by the iron chelator deferoxamine in a rodent intracerebral hemorrhage model [110]. More basic research is needed to confirm the role of iron in SAH.

## 6. Management and Treatment

Although a growing number of studies have focused on white matter injury after SAH, all treatment and management targeting WMI are still limited to basic research, and there is no specific treatment for human WMI in SAH. According to the mechanisms of WMI in SAH, there are potential treatments targeting WMI (Table 1).

As mentioned above, acute and chronic hydrocephalus is a common complication after SAH and could damage white matter fibers in deeper areas of the brain. Surgical removal may be an effective treatment for hydrocephalus after SAH, as it can relieve nerve compression, lower intracranial pressure, and improve patient outcomes. The main surgical methods include external ventricular drainage for acute hydrocephalus and permanent shunt diversion for chronic hydrocephalus [111–114].

Delayed cerebral ischemia is characteristic of SAH and represents a significant cause of poor functional outcomes. White matter is highly vulnerable to ischemia than gray matter. Delayed cerebral ischemia was mainly thought to be caused by cerebral vasospasm [115]. Experimental studies and clinical research have suggested that calcium antagonists can prevent or reverse vasospasm and reduce the risk of poor outcomes and secondary ischemia after SAH [116]. Most guidelines recommend nimodipine for vasospasm to improve the prognosis of patients with aneurysmal SAH [117]. In addition, a randomized controlled trial showed that erythropoietin may improve patient outcomes via decreasing the severity of vasospasm [118].

Oligodendrocytes and axonal plasticity play important roles in maintaining the structure and function of white matter. Therefore, interventions targeting oligodendrogenesis and axonal plasticity might improve behavioral outcomes after SAH. NMDAR antagonist memantine has shown some effectiveness in the treatment of vascular dementia in the clinical setting [119]. The therapeutic effects of memantine might be through mitigating oligodendrocyte damage to attenuate white matter injury [120, 121]. Moreover, there are a variety of drugs that promote remyelination or impedance demyelination in preclinical stages. And relevant clinical studies need to be further conducted.

At present, most of the mechanistic studies related to BBB disruption, neuroinflammation, iron deposition, and so on are still at the stage of laboratory research. And the clinical results are still insufficient to support the effectiveness of mechanism-related drugs and treatment for WMI after SAH. Further investigations are required to directly address these issues.

## 7. Perspective and Conclusion

As a consequence, WM is exquisitely vulnerable to SAH, and WMI results in profound cognitive dysfunction, emotional disorders, and so on after SAH. Most studies have emphasized GM and overlooked the critical role of WM in damage and recovery after SAH. However, long-lasting neuroprotection cannot be attained without parallel protection of WM. Protecting the integrity and connectivity of WM is expected to facilitate the rehabilitation of WM networks and improve SAH prognosis. Therefore, future SAH therapies need to be designed to be inclusive of both GM and WM.

The majority of hypotheses and mechanisms of WMI after SAH have been studied and verified in animal models, and plenty of basic research had demonstrated many therapeutic targets and medicine for SAH-induced WMI, such as MMP-9, LCN2, PTEN, MCT1, COG1410, and MLT [26, 41, 90, 92, 98, 122]. But it remains poorly investigated in SAH patients. There are major differences between human and animal models, and the human condition after SAH is far more complex than rodent SAH models. Therefore, more mechanistic studies need to be performed in the clinical setting.

SAH is a complex process involving multiple intertwined mechanisms. Treatments of SAH need to target multiple underlying mechanisms over time and space. Although GMI and WMI after SAH share some common characteristics, WMI exhibits unique properties. Furthermore, axons, astrocytes, and oligodendrocytes, along with progenitor cells, surrounding microglia, and vasculature constitute a highly complex framework for WM-targeting strategies. Multiple cell types and intercellular signaling cascades contribute to the maintenance of WM integrity and connectivity [123]. Thus, further investigations of WMI should emphasize cellular networks rather than solely focusing on a single cell type.

## Figures and Tables

**Figure 1:** Characteristics of white matter.

**Figure 2:** Pathological mechanisms of white matter injury after subarachnoid hemorrhage.

**Figure 3:** Schematics for the pathogenic factors of white matter injury after subarachnoid hemorrhage. ICP: intracranial pressure; BBB: blood-brain barrier.

**Table 1:** Management and treatment of white matter injury after subarachnoid hemorrhage.

Stage	Strategy	Management and treatment
Clinical setting	Alleviating hydrocephalus	External ventricular drainage
		Permanent shunt diversion
	Reducing vasospasm	Nimodipine
		Erythropoietin
	Preventing vascular dementia	NMDAR antagonist memantine

Laboratory research	Alleviating BBB disruption	LCN2 knockout
	Reducing neuroinflammation	Microglial depletion by CLP pretreatment Promote M2 microglial polarization by COG1410
	Protection of oligodendrocyte and OPC	LCN2 knockout for reducing injury LCN2 knockout for OPC differentiation Nexilin for regulating OPC migration
		MLT for reducing apoptosis in oligodendrocytes
